# The Value of a Management Plan Based on Risk Factors for Cerebral Infarction Patients with Cerebral Hemorrhage

This article has been retracted.

**DOI:** 10.1155/2022/8635487

**Published:** 2022-04-08

**Authors:** Jinfeng Dang, Jieting Li, Haixia Li, Gaoyan Pian, Zhizhuan Guo

**Affiliations:** Shanxi Bethune Hospital Department of Neurology, Taiyuan 030032, China

## Abstract

Cerebral infarction is a neurological disease related to abnormal blood supply to brain tissue. Patients are mainly men between the ages of 50 and 60 years old. In order to explore the value of risk factor-based management programs for preventing hemorrhagic conversion in patients with cerebral infarction, this paper uses single and multifactor methods to analyze the risk factors of cerebral hemorrhage transformation after cerebral infarction and formulate risk factor-based management plans. 240 cases of cerebral infarction who were admitted to our hospital in the past 2 years were evenly divided into an intervention group (intervention based on risk factors) and a routine group (regular care mode) by a simple randomized method. Cerebral hemorrhage is observed in both groups. We assessed the stroke scale of the National Institutes of Health (NIHSS) score. The development of risk factor-based management plans for patients with acute cerebral infarction during the treatment period has important clinical significance for reducing the incidence of hemorrhagic conversion in patients and promoting the recovery of neurological function.

## 1. Introduction

Cerebral infarction is a neurological disease related to abnormal blood supply to brain tissue [1]. Patients are mainly men between the ages of 50 and 60 years old. In the early stages of the disease, patients usually have no prodrome. Some patients may experience transient dizziness and limb numbness, and after onset, patients may develop hemiplegia, aphasia, cerebral hernia, coma, and other symptoms [2]. After the onset of cerebral infarction, patients with cerebral ischemia may experience bleeding in the area, clinically known as hemorrhagic conversion. Investigations have shown that 9% of patients with cerebral infarction may experience hemorrhagic conversion [3]. After hemorrhagic transformation occurs, the patient's condition further deteriorates, which seriously negatively affects the patient's recovery efficiency and directly endangers the patient's life. Therefore, it is of great importance to determine the risk factors for hemorrhagic conversion in patients with cerebral infarction and perform targeted management to prevent and treat hemorrhagic conversion [4].

In order to examine the efficacy of risk factor-based management programs for preventing hemorrhagic conversion in patients with cerebral infarction, a total of 87 patients with hemorrhagic conversion in cerebral infarction were selected for this study. The development of risk factor-based management plans for patients with acute cerebral infarction during the treatment period has important clinical significance for reducing the incidence of hemorrhagic conversion in patients and promoting the recovery of neurological function.

## 2. Data Collection and Intervention Methods

For the first part of our study, we retrospectively enrolled 87 cases of cerebral infarction complicated by cerebral hemorrhage conversion (case group) and 90 cases of cerebral infarction without cerebral hemorrhage conversion (control group) who were admitted to our hospital. The risk factors for cerebral infarction complicated by intracerebral hemorrhage transformation are analyzed using univariate and multivariate methods, and targeted intervention measures are formulated according to the risk factors. A total of 240 patients with cerebral infarction who were admitted to our hospital in the past 2 years are divided into two groups: the intervention group (intervention based on risk factors; 120 cases) and the routine group (routine management mode; 120 cases), using a simple randomized method. The inclusion criteria are as follows: (1) met to the diagnostic criteria for cerebral infarction [5, 6]; (2) aged between 19 and 79 years; and (3) and received treatment in our hospital. The exclusion criteria are as follows: (1) patients diagnosed by imaging with lacunar cerebral infarction and white matter laxity [7]; (2) previous history of cerebral hemorrhage; (3) patients with respiratory cycle or brain stem infarction failure; (4) the use of anticoagulants and other related drugs before cerebral infarction; and (5) history of intracranial tumor or other malignant tumors. The study protocol was approved by the Medical Ethics Committee of our institution, and informed consent was signed by the patients' family members before intervention.

### 2.1. Data Collection

Age, sex, body mass index (BMI), smoking, drinking, combined diabetes, hypertension, coronary heart disease, history of atrial fibrillation, NIHSS score at admission, cerebral infarction site, whether it is a large-area cerebral infarction, antiplatelet aggregation therapy, anticoagulation therapy, thrombolytic therapy, serum triglyceride (TG), total cholesterol (TC), high-density lipoprotein cholesterol (HDL-C), low-density lipoprotein cholesterol (LDL-C), platelet count (PLT), coagulation time (PT), fibrinogen (Fib), brain volume (rCBV), cerebral blood flow (rCBF), and mean passage time (MTT) are collected for the case and control groups.

### 2.2. Intervention Methods

The routine group (routine intervention and nursing mode): patients are given medication guidance, health knowledge, and psychological intervention at the same time.

The intervention group (risk factor-based management program interventions): (1) antiatrial fibrillation intervention: The ECG status of patients is closely observed, the causes of atrial fibrillation are analyzed, and targeted treatments are conducted, such as antihyperthyroidism, anti-infection, and electrolyte balance. We monitored the patient's blood oxygen level. As hypoxia may cause or aggravate atrial fibrillation, when arterial blood oxygen partial pressure is less than 60 mmHg, an oxygen inhalation operation is performed while simultaneously monitoring the blood oxygen status. We also conducted psychological counseling for patients to help eliminate negative emotions and improve confidence in the treatment. (2) Coagulation function intervention: patients' coagulation function is closely monitored, anticoagulation therapy is conducted according to individual patient circumstances, and at the same time, patients are instructed to rest and relieve their emotions. Patients are recommended to follow a diet that is light and avoid too much oil, spicy, and sweet foods, and supplement high amino acid foods, which could aid in maintaining the body's weak acid level to reduce intracranial hematoma symptoms. (3) Intervention of ischemia-reperfusion injury: ischemia-reperfusion injury is closely related to hemorrhagic conversion in patients with cerebral infarction. To reduce the incidence of ischemia-reperfusion injury in cerebral infarction ischemia, methylprednisolone shock therapy should be performed according to the patient's condition. (4) Patients are treated with thrombolysis to restore blood oxygen supply to the infarct area. Body temperature is monitored, the causes of abnormal body temperature are analyzed, and patients showing signs of infection are treated with antibiotics. Brain edema and brain hernia are common complications of large-area cerebral infarction, and medical staff should closely monitor patients' vital signs, such as gaze paralysis, periodic breathing, papillary edema, and other manifestations, and suspected cerebral hernia. At this time, medical staff should immediately elevate the upper torso of the patient, be careful to protect the jugular vein when the head and neck are raised to avoid jugular vein compression, and administer intravenous mannitol as appropriate [8]. The infarct area and edema status of the patients are observed by imaging, and surgery is required in severe cases [9]. (5) Rehabilitation intervention: patients are given passive exercises for the distal joints, such as palm, plantar, elbow, and knee, once a day for 15 min [10]. Joint movement is gentle and slow to avoid joint damage caused by violent massage. Patients are encouraged to actively communicate and improve their language functions [11]. For patients with pronunciation difficulties, medical staff conducted pronunciation training once a day for 10 min. (6) Daily intervention: the patient's self-care ability is usually insufficient; thus, medical staff aid patients with defecation, urine care, and regularly change the bedding [12]. Long-term bedridden patients require turning every 2 h, and the compression side is massaged for 10 minutes to promote blood circulation. The patients are asked to drink more water, and the medical staff regularly cleaned the patients' urethral openings to avoid urinary system infection.

SPSS software (version 21.0; IBM, New York, USA) is used for data analyses. In our study, the Fib, CBV, CBF, MTT, and other measurement indexes are all normally distributed and are expressed as ($\bar{x}\pm s$). A *t*-test is used for intergroup analysis, the *χ*^2^ test is used for intergroup analysis of enumeration data, and a logistic regression model is used for multivariate analysis (test level *α* = 0.05).

## 3. The Experimental Results

### 3.1. Single Factor Analysis

There is no statistical difference in age, gender, BMI, smoking, drinking, hypertension, coronary artery disease, NIHSS score at admission, cerebral infarction site, antiplatelet aggregation therapy, anticoagulation therapy, thrombolytic therapy, serum TG, TC, HDL-C, LDL-C, PLT, and PT between the case and control groups (*P* > 0.05). Comparison of the combined diabetes, atrial fibrillation history, whether it is a large area cerebral infarction, Fib, CBV, CBF, and MTT between the case and control groups showed statistically significant differences (*P* < 0.05).  Table 1 shows the single factor analysis results.

### 3.2. Logistic Multivariate Analysis

Diabetes, history of atrial fibrillation, large-area cerebral infarction, Fib, rCBV, rCBF, and MTT are used as independent variables. The logistic regression model showed that cerebral infarction combined with atrial fibrillation, increased Fib, increased MTT, and large-area cerebral infarction are independent risk factors for cerebral hemorrhagic conversion (*P* < 0.05). Increased rCBV and rCBF values can reduce the occurrence of hemorrhage in patients with a high probability of hemorrhagic conversion (*P* < 0.05).  Table 2 shows the logistic multivariate analysis results.

### 3.3. Comparison of Baseline Data between the Intervention and Routine Groups

Statistical analysis showed that there were no statistically significant differences in age, sex, BMI, smoking, drinking, hypertension, coronary artery disease, NIHSS score at admission, cerebral infarction site, antiplatelet aggregation therapy, anticoagulation therapy, thrombolytic therapy, and baseline data between the intervention and routine groups (*P* > 0.05).  Table 3 presents a comparison of baseline data between the intervention group and the routine group.

### 3.4. Comparison of the Incidence of Hemorrhagic Conversion between the Intervention and Routine Groups

Twenty-eight days after treatment, seven cases (5.83%) in the intervention group showed higher hemorrhagic conversion than the 19 cases (15.83%) in the routine group, and the difference is statistically significant (*P* < 0.05).  Table 4 displays a comparison of the incidence of hemorrhagic conversion between the two groups after 28 days of treatment.

### 3.5. Changes in NIHSS Scores in the Intervention and Routine Groups after 28 days of Treatment

Before treatment, there is no significant difference in the NIHSS scores between the intervention and routine groups (*P* > 0.05). After 14 days and 28 days of treatment, the NIHSS scores are lower in the intervention group than in the routine group (*P* < 0.05).  Table 5 shows changes in NIHSS scores of the intervention and routine groups after 28 days of treatment.

## 4. Experimental Result Analysis

Hemorrhagic conversion is a common complication, leading to deterioration in the condition of patients with cerebral infarction. Studies have shown that even a low hemorrhagic transition can lead to increased brain tissue damage and poor prognosis. However, the clinical mechanism of hemorrhage transformation in patients with cerebral infarction is uncertain, and some studies confirmed that it may be related to dysfunction of endothelial cells in the infarct, causing changes in vascular permeability; thus, leading to exudation of red blood cells, which may also be related to blood reperfusion injury and collateral circulation of the infarct. In this study, to improve the prognosis of hemorrhage transformation in patients with cerebral infarction, the risk factors of patients with hemorrhagic conversion were analyzed, and risk management was carried out.

We observed significant differences between the case and control groups in combined diabetes, atrial fibrillation history, large-area cerebral infarction, Fib, CBV, CBF, and MTT, suggesting that these factors are related to cerebral infarction with hemorrhagic conversion. The logistic regression model showed that cerebral infarction combined with atrial fibrillation, increased Fib, increased MTT, and large-area cerebral infarction are independent risk factors for cerebral hemorrhagic conversion (*P* < 0.05). Increased rCBV and rCBF values can reduce the occurrence of hemorrhage in patients with a probability of conversion. Atrial fibrillation can cause blood clots in the walls of the atria to disengage and enter the circulatory system. Once these clots enter the brain, they can cause cerebral embolism because the cardiac thrombosis volume is large. Large-area cerebral infarction is easily caused by cerebral obstruction. In addition, the large area of tissue hypoxia mediated by a large-area cerebral infarction will lead to intima injury in this area, induce a change in permeability, and trigger erythrocyte extravasation bleeding conversion. Meanwhile, the cells in the cerebral infarction foci will also swell due to hypoxia, which leads to compression and injury of the peripheral microvessels, resulting in the appearance of spots or patches of small bleeding foci. An increase in the Fib value indicates that the patient's blood is in a hypercoagulable state, which will lead to an increase in the thrombosis rate, an increase in the cerebral infarction rate, and muscle infarction area, which further increases the risk of hemorrhagic conversion. An increase in the MTT value indicates an increased risk of ischemia-reperfusion injury, and ischemia-reperfusion injury results in the destruction of the blood-brain barrier in patients with coinflammation, damages the function of the cerebrovascular self-regulation system, and finally causes hemorrhagic conversion. Improvement of rCBV and rCBF can restore the blood supply of the infarct to some extent, and therefore restore the nerve and vascular functions in the area and improve the self-regulation ability of the blood vessels; thus, reducing the related bleeding risk.

With regards to the intervention effect, after 14 days and 28 days aftertreatment, NIHSS scores in the intervention group were lower than those in the routine group, indicating that the risk factor-based management regimen had a significant advantage in promoting the recovery of cerebral nerve function in patients with cerebral infarction and hemorrhagic conversion. Meanwhile, within 28 days after treatment, 19 patients (15.83%) in the intervention group developed hemorrhagic conversion, compared to seven patients (5.83%) in the routine group, suggesting that risk factor-based management plans can effectively reduce the complication rate of hemorrhagic conversion, thus improving the prognosis of patients. Risk factor-based management plans are highly pertinent and can handle and determine the potential risk of hemorrhagic transition in advance, which can reduce the incidence of hemorrhage transformation in patients with cerebral infarction as well as damage to brain tissue, thus improving nerve function.

## 5. Conclusion

In conclusion, according to the risk factors of hemorrhagic conversion in patients with cerebral infarction, the development of risk factor-based management plans to intervene in patients with acute cerebral infarction during the treatment period has important clinical significance for reducing the incidence of hemorrhagic conversion in patients and promoting the recovery of neurological function.

It is important to note that some studies verified that the treatment regimen used in patients with cerebral infarction may also lead to hemorrhagic conversion; thrombolysis-mediated blood flow recirculation may lead to focal vascular hemorrhage with structural damage, so thrombolysis therapy for cerebral infarction patients should strictly grasp the timing and indications. However, this conclusion was not verified in our study and may need to be confirmed by subsequent research.

## Figures and Tables

**Table 1:** Single factor analysis results.

Normal information	Case group (*n* = 87)	Control group (*n* = 90)	*t*/*χ*^2^	*P*
Age (years)	68.2 ± 7.5	67.0 ± 6.8	1.116	0.266
BMI (kg/m^2^)	24.1 ± 2.0	23.8 ± 2.5	0.880	0.380
Gender (%)				
Male	48 (55.17)	56 (62.22)	0.907	0.341
Female	39 (44.83)	34 (37.78)		
Smoking (%)				
Yes	29 (33.33)	38 (42.22)	1.486	0.223
No	58 (66.67)	52 (57.78)		
Drinking (%)				
Yes	22 (25.29)	29 (32.22)	1.037	0.308
No	65 (74.71)	61 (67.78)		
Diabetes (%)				
Yes	35 (40.23)	20 (22.22)	6.698	0.010
No	52 (59.77)	70 (77.78)		
Hypertension (%)				
Yes	43 (49.43)	48 53.33)	0.270	0.603
No	44 (50.57)	42 (46.67)		
Coronary heart disease (%)				
Yes	18 (20.69)	11 (12.22)	2.315	0.128
No	69 (79.31)	79 (87.78)		
History of atrial fibrillation (%)				
Yes	24 (27.59)	11 (12.22)	6.582	0.010
No	63 (72.41)	79 (87.78)		
Cerebral infarction site (%)				
Cortex	45 (51.72)	37 (41.11)	2.004	0.157
Subcortical	42 (48.28)	53 (58.89)		
Massive cerebral infarction (%)				
Yes	54 (62.07)	36 (40)	8.621	0.003
No	33 (37.93)	54 (60)		
Platelet aggregation therapy (%)				
Yes	39 (44.83)	31 (34.44)	1.995	0.158
No	48 (55.17)	59 (65.56)		
Anticoagulant therapy (%)				
Yes	49 (56.32)	39 (43.33)	2.985	0.084
No	38 (43.68)	51 (56.67)		
Thrombolytic therapy (%)				
Yes	13 (14.94)	7 (7.78)	2.266	0.132
No	74 (85.06)	83 (92.22)		
NIHSS score at admission (scores)	13.12 ± 3.18	12.59 ± 2.77	1.183	0.238
TG (mmol/L)	1.64 ± 0.28	1.59 ± 0.25	1.254	0.211
TC (mmol/L)	4.93 ± 0.45	4.80 ± 0.49	1.837	0.068
HDL-C (mmol/L)	1.10 ± 0.16	1.15 ± 0.18	−1.951	0.053
LDL-C (mmol/L)	3.28 ± 0.57	3.16 ± 0.53	1.451	0.149
PLT (×10^9^/L)	189.6 ± 22.7	195.8 ± 25.3	−1.714	0.088
PT (s)	15.9 ± 1.2	15.7 ± 1.4	1.019	0.310
Fib (g/L)	3.95 ± 0.78	3.52 ± 0.71	3.838	≤0.001
rCBV (100 g/min)	9.45 ± 2.61	28.71 ± 6.33	−26.299	≤0.001
rCBF (ml/100g)	1.54 ± 0.46	3.06 ± 0.95	−13.474	≤0.001
MTT (s)	9.56 ± 1.84	7.84 ± 1.88	6.149	≤0.001

**Table 2:** Logistic multivariate analysis results.

Index	*b*	SE	Walds	*P*	OR	95% CI	
Diabetes	0.498	0.337	2.184	0.226	1.645	0.850	3.185
History of atrial fibrillation	0.471	0.196	5.775	0.018	1.602	1.091	2.352
Massive cerebral infarction	0.582	0.267	4.751	0.042	1.790	1.060	3.020
Fib	0.264	0.117	5.091	0.037	1.302	1.035	1.638
rCBV	−0.773	0.354	4.768	0.042	0.462	0.231	0.924
rCBF	−0.330	0.186	3.148	0.108	0.719	0.499	1.035
MTT	0.253	0.297	0.726	0.424	1.288	0.720	2.305
Constant term	1.209	0.482	6.292	0.008	3.350	1.302	8.617

**Table 3:** Comparison of baseline data between intervention group and routine group.

Normal information	Intervention group (*n* = 120)	Routine group (*n* = 120)	*t*/*χ*^2^	*P*
Age (years)	66.8 ± 8.0	67.4 ± 6.1	−0.653	0.514
BMI (kg/m^2^)	23.8 ± 2.0	23.5 ± 2.7	0.978	0.329
NIHSS score at admission (scores)	13.55 ± 2.94	12.87 ± 2.80	1.835	0.068
Gender (%)				
Male	65 (54.17)	73 (60.83)	1.091	0.296
Female	55 (45.83)	47 (39.17)		
Smoking (%)				
Yes	43 (35.83)	36 (30.00)	0.925	0.336
No	77 (64.17)	84 (70.00)		
Drinking (%)				
Yes	39 (32.50)	45 (37.50)	0.659	0.417
No	81 (67.50)	75 (62.50)		
Diabetes (%)				
Yes	54 (45.00)	63 (52.50)	1.351	0.245
No	66 (55.00)	57 (47.50)		
Hypertension (%)				
Yes	65 (54.17)	57 (47.50)	1.067	0.302
No	55 (45.83)	63 (52.50)		
Coronary heart disease (%)				
Yes	18 (15.00)	24 (20.00)	1.039	0.308
No	102 (85.00)	96 (80.00)		
History of atrial fibrillation (%)				
Yes	15 (12.50)	23 (19.17)	2.001	0.157
No	105 (87.50)	97 (80.83)		
Cerebral infarction site (%)				
Cortex	63 (52.50)	72 (60.00)	1.371	0.242
Subcortical	57 (47.50)	48 (40.00)		
Massive cerebral infarction (%)				
Yes	48 (40.00)	56 (46.67)	1.086	0.297
No	72 (60.00)	64 (53.33)		
Platelet aggregation therapy (%)				
Yes	48 (40.00)	59 (49.17)	2.041	0.153
No	72 (60.00)	61 (50.83)		
Anticoagulant therapy (%)				
Yes	58 (48.33)	51 (42.50)	0.824	0.364
No	62 (51.67)	69 (57.50)		
Thrombolytic therapy (%)				
Yes	49 (40.83)	57 (47.50)	1.081	0.298
No	71 (59.17)	63 (52.50)		

**Table 4:** Comparison of the incidence of hemorrhagic conversion between the two groups after 28 days of treatment.

Group	*n*	No bleeding transformation	Hemorrhagic transformation
Intervention group	120	7 (5.83)	113 (94.17)
Regular group	120	19 (15.83)	101 (84.17)
*X* ^2^		6.211	
*P*		0.013	

**Table 5:** Changes in NIHSS scores of the intervention and routine groups after 28 days of treatment ($\bar{x}\pm s$, scores).

Group	*n*	Before therapy	After 14 days of treatment	After 28 days of treatment
Intervention group	120	13.55 ± 2.94	7.96 ± 1.88	4.41 ± 1.50
Regular group	120	12.87 ± 2.80	8.61 ± 2.24	4.84 ± 1.78
*X* ^2^		1.835	−2.435	−2.024
*P*		0.068	0.016	0.044

## Data Availability

The simulation experiment data used to support the findings of this study are available from the corresponding author upon request.
